RETRACTED

# The Association of COVID-19 Pandemic Stress With Health-Related Quality of Life in the Kingdom of Saudi Arabia: A Cross-Sectional Analytical Study

**DOI:** 10.3389/fpubh.2021.600330

**Published:** 2021-03-05

**Authors:** Manal Mohammed Hawash, Amani Hamad Alhazmi, Wagida Wafik, Khursheed Muzammil, Sakeena Mushfiq, Hala Awad Ahmed

**Affiliations:** ^1^Department of Public Health, College of Applied Medical Sciences, Khamis Mushayt, King Khalid University, Abha, Saudi Arabia; ^2^Department of Gerontological Nursing, College of Nursing, Alexandria University, Alexandria, Egypt; ^3^Department of Community Health Nursing, College of Nursing, Zagazig University, Zagazig, Egypt

**Keywords:** COVID-19, stress, health-related quality of life, lockdown, pandemic, PSS-10

## Abstract

**Background:** There is a global disaster since WHO declared Covid-19 as a pandemic. With the increase in cases & mortality rate, various health issues viz., stress, mental disorders and altered health-related quality of life have been noted as a result of pandemic and lockdowns. This study aimed to assess the association of COVID-19 pandemic stress with health-related quality of life in the Kingdom of Saudi Arabia.

**Methodology:** It was a cross-sectional analytical study. Subjects included 878 citizens and residents of Saudi Arabia aged 18 years and above. Convenience, non-probability sampling technique was used. A web-based, self-administered, electronic questionnaire in Arabic language having three sections; Sociodemographic & clinical profile, Standard PSS-10, and Standard SF-12 was used as the study tool and distributed through various social media means. The study period was of 2 months. Data were analyzed using SPS version 25. Descriptive statistics, Pearson's correlation coefficient, independent sample *t*-test and the one-way analysis of variance (ANOVA) were employed for suitable statistical analysis.

**Results:** Almost two-thirds of the subjects were between the age of 18 to < 40 and majority (74.1%) being females. Majority (83.0%) reported as having no chronic diseases, and 69.5% had no contact history with COVID-19 cases. The mean of MCS & PCS was (32.34 ± 25.30) & (41.65 ± 11.82), respectively. Majority (67.6%) had a moderate level of COVID-19 stress. A significant negative relationship between total stress scores and HRQOL domains was observed.

**Conclusion:** Majority subjects had a moderate level of stress related to COVID-19 lockdown. Stress during COVID-19 has a significant negative association with both physical and mental HRQOL in which MCS was significantly lower than PCS. It is recommended to evaluate the effectiveness of stress management program and follow a holistic approach.

RETRACTED

## Introduction

Nowadays, the world-wide scientific attention has recently focused on novel coronavirus disease 2019 (COVID-19) The World Health Organization (WHO) has stated that COVID-19 is considered as a major public health disaster which has rigorously affected the world and poses an urgent and severe global health threat. Since WHO has declared COVID−19 as a pandemic, humanity becomes exceptionally vulnerable (1). The clinical manifestations of COVID-19 vary from an asymptomatic to severe infectious disease. The confirmed cases of COVID - 19 are rapidly increased with significant mortality rate causing various deleterious health problems such as stress, fear of the unknown, anxiety and depression both in health care personnel and in the general population (2).

COVID-19 is a new viral disease which influences humans and spreads promptly from human to human via respiratory droplets. The transmission of this new coronavirus 2019 is exponentially increased all over the world. As there is no specific treatment modality and currently vaccine is being administered in a phase wise manner, still the required emphasis is to keep populations aware of the widespread preventive protocol. These preventive protocols are the only reliable solution to control the transmission of this viral infection by wearing face masks, extensive hygiene precautions, and social distancing. Accordingly, numerous nations have implemented firm quarantine and prohibited the people gatherings to breakdown the exponential COVID-19 spread curve, which in turn hampers the deadly consequences of this contagious disease (3). The first COVID-19 case in Saudi Arabia was reported on 2nd March 2020. Since then, many rapid and crucial preventive quarantine measures have been applied to lessen daily infected cases and death numbers (4). As of 28th of January 2021, currently confirmed cases in Saudi Arabia stands at 367,276 with 6,366 deaths, which indicates less transmission and consequently less mortality (5).

Many people's emotional and mental health become at risk as a result of these lockdown measures which vary from compulsory quarantine to voluntary self-isolation. Overall, the self-imposed isolation and lockdown has an enormous effect, causing significant psychological strain that influences many aspects of people's lives, and subsequently leading to multiple psychological disorders (6). A study conducted in China showed that the unknown fear could trigger mental problems like depression, anxiety, and deviant risk behaviors such as tobacco, and alcohol consumption (7). During the lockdown period, people staying at home are expected to have higher levels of stress especially among individuals with chronic illness, and multiple comorbidities. As well, the elders remain anticipated to be psychologically more susceptible to mental stress as the result of the COVID-19 pandemic than adults who have self-perceived invulnerability or optimistic bias (3). Study conducted in China by Qiu et al. also confirmed that almost 35% of subjects exhibited emotional distress (8). Similarly, a recent survey revealed that 53.8% of respondents assessed COVID-19 outbreak psychological impact as moderate or severe; 8.1% documented moderate to severe levels of stress; 28.8 and 16.5% of the study subjects showed moderate to severe anxiety symptoms, and depressive symptoms, respectively (9).

RETRACTED

Numerous individuals are facing the stress of varying types and levels because of the COVID −19 lockdowns. Therefore, the COVID-19 outbreak is considered an irrepressible traumatic life event resulting in hampering the Quality of life (QOL) in general & health-related quality of life (HRQoL) in particular. HRQoL is a multidimensional concept defined as the way by which the individuals estimated his/her mental, physical, emotional and social domains of well-being (10). Flint et al. conducted their study in Canada and reported that COVID-19 has direct and indirect adverse physical and psychosocial health consequences (11). Due to the COVID-19 containment measures, the daily routine life of all human beings have been affected, and ultimately has an association with their health and well-being globally in all spheres. Despite the significance of the stress-related COVID – 19, data are lacking about its association with health-related quality of life. Thus, there is an utmost need to study the association of stress-related to COVID – 19 with Health-Related Quality of Life (HR-QOL) to assist the policymakers in designing adequate specific preventive interventions/measures to avoid hampering of Health-Related Quality of Life (HR-QOL) among masses (12). COVID-19 pandemic plays a vital role in exerting psychological and physiological stress on common men & women, social organizations and businesses globally. It may have far-reaching implications for HRQoL into the future. COVID - 19 affects body systems and is associated with the psychological status of those either having chronic illnesses or not also. Considering the current scenario of COVID-19, it becomes relevant for the researchers to address the factors that may correlate with HRQoL.

The whole world is witnessing similar disastrous conditions, but the current study has been designed as an initiative in the Kingdom of Saudi Arabia. Therefore, this study aimed to assess the association of COVID-19 pandemic stress with health-related quality of life, KSA along with two objectives viz., (a) To determine the level of perceived Stress during COVID-19&HR-QOL status among the respondents during pandemic lockdown era, (b) To identify the association between perceived COVID −19 stress level & HR-QOL (c) to identify factors associated with COVID−19 stress among the participants during the pandemic lockdown era. The respondents' socio-demographic characteristics (education, occupation, family income) and self-reported preexisting chronic conditions (diabetes, cardiovascular & respiratory diseases) were included in determining their association with COVID−19 stress.

RETRACTED

## Methodology

### Study Design and Sample

A cross-sectional analytical study was conducted among all the citizens and residents aged 18 years and above, living all over the Kingdom of Saudi Arabia during COVID – 19 pandemic lockdowns. With reported internet usage in KSA at an impressive 93% in Jan 202 (13), self-reported online questionnaires were chosen as a data collection tool so that outreach could be maximized in a short span of time. A convenience, non-probability sampling technique was used to recruit the study participants. A minimum representative sample of 664 was calculated by online software RAOSOFT (14) using a margin of error of ±5%, a confidence level of 99%, a 50% response distribution with total population 34,218,169. As the first step of data collection, various popular social media platforms were chosen, such as WhatsApp, Twitter. Among these, several specific groups of students, teachers, mothers etc. were identified randomly, and the link for the web-based electronic questionnaire (https://forms.gle/MpzBKQgAvW8ux6MM8) was shared with them, with requests to distribute further to their family members, colleagues, friends, and neighbors etc. Data collection was continued for a period of 1 month from 01 June to 30 June 2020, ending few days after the lifting off of quarantine restrictions in KSA (i.e., 21/6/2020). At the end of the data collection period, a total of 878 responses was received and analyzed via online communication network programs.

### Study Tool/Measurements

Data were collected using a web-based, self-administered, electronic questionnaire in the Arabic language. It comprised of three sections. The first section assessed the socio-economic, demographic profile and clinical data of the respondents comprising age, sex, nationality, marital status, level of education, place of residence, type of occupation (related to the medical field or not), financial status and presence of chronic illness (diabetes, cardiovascular & respiratory diseases etc). Apart from that, participants were also asked if he/she was either COVID - 19 patient or has had close contact with COVID - 19 cases.

RETRACTED

The second section consisted of ten items measuring the perception of stress using pre-designed and pre-tested Perceived Stress Scale (PSS-10). The PSS-10 was used to measure the level/ extent to which situations such as COVID - 19 pandemic in one's life was perceived. This 10-item PSS version was developed by Cohen et al. (15). Arabic version of the PSS-10 questionnaire was used in this study. It is a reliable, valid tool which was translated from English to the Arabic language by Almadi et al. (16). The Cronbach's alpha coefficients was 0.80 for overall 10-items PSS scale. This scale contains ten items regarding the feelings and thoughts of the respondents during the last month from the day of administering the tool. It is a 5-point Likert scale in which each item was scored from 0 (never) to 4 (very often). The total score of this scale ranged from 0 to 40 in which higher scores displaying higher perceived COVID19 stress. Scores ranging from 0 to 13 is reflected as low perceived stress. Scores ranging from 14 to 26 is considered moderate perceived stress, whereas scores ranging from 27 to 40 is revealed as high perceived stress.

The third section included twelve items Short Form Health Survey (SF-12), which is a multipurpose valid generic measure of health status/outcomes. It was used to examine subjects' HRQoL, and to monitor the health of both general and specific population. The 12-items SF version was developed by Ware et al. (17). It includes 12 questions measuring eight health concepts/dimensions; two questions for physical functioning, two questions for role limitation due to physical health problems, one question for bodily pain, one question for general health, one question for vitality, one question for social functioning, two questions for role limitation due to the emotional problems, and two questions for mental health. This study has used the Arabic version of the SF-12 questionnaire, translated from English, by Al-Shehri et al. (18). Overall reliability of Arabic Version was found to be good, at Chronbach alpha = 0.84 (18). Response categories for items ranged from two- to six-point scales, and raw scores for items range from 1 to 6. The Quality Metric Health Outcomes Scoring Software 2 was used after recording in order to transform the raw scores of each scale items without standardization or weighing to calculate subscales scores, each ranging from 0 (the worst) to 100 (the best). Then a norm-based scoring algorithm analytically derived from US data of general population survey was applied. The norm-based scores were attained by applying the succeeding formula; Transformed score for each scale= (original score of the scale – the lowest score possible origin)/(range of possible scores for the original scale)^*^100. To calculate PCS, and MCS components summary scores, it has been assumed a mean of 50 and an SD of 10 based on US-derived summary scores (17).

RETRACTED

### Statistical Methods

The collected data was checked twice for its correctness & completeness. The data was coded and also analyzed for suitable statistical significance with the help of Microsoft Excel and Statistical Package for Social Sciences (SPSS)version 25. Descriptive statistics as frequency, mean, standard deviation, median, and coefficient of variation were used to describe different quantitative and qualitative variables. One –sample Kolmogorov Smirnov test was used to be assured that the SF12 domains had a normal distribution. Pearson coefficient is used to correlate between two normally distributed quantitative variables. Independent-sample *t*-test is used to determine whether there are any statistically significant differences between the means of two independent groups. The one-way analysis of variance (ANOVA) has been used to know whether there are any statistically significant differences between the means of two or more independent variables or not. The level of significance selected for this study was *p*-value equal to or <0.05.

### Ethical Considerations and Consent

The Research Ethics Committee of King Khalid University has already approved the study. Informed consent was taken before data collection. Confidentiality of the collected data was ensured.

## Results

Table 1 shows the socio-economic and demographic profile of the study participants. Almost two thirds (64.4%) of the participants were between the age of 18 and <40 and only 2.6% of them aged ≥60. The majority (74.1%) of the studied subjects were females, and nearly two-thirds (62.4%) of them were married. The majority (85.1%) of the participants were Saudi citizens, and (82.8%) had graduation or postgraduate education. Almost half (46.5%) of the subjects were from the Asir region, whereas 0.6% of the participants were from the Northern Border region. Out of the total participants, 48.9% were government employees, and 2.2% were non-government employees. Of the total sample, about half (49.4%) of the participants reported that their economic status was sufficient.

**Table 1:** Socio-demographic characteristics of the study participants (*N* = 878).

**Socio-demographic variables**	**Categories**	**No**.	**(%)**
Age	18 to <40	565	64.4
	40 to <60	290	33.0
	≥60	23	2.6
Sex	Male	227	25.9
	Female	651	74.1
Nationality	Saudi	747	85.1
	Non-Saudi	131	14.9
Educational level	Primary education	24	2.7
	Secondary education	127	14.5
	Graduation/Postgraduation	727	82.8
Marital status	Married	548	62.4
	Unmarried	330	37.6
Provinces of Residence	Asir	408	46.5
	Makkah	252	28.7
	Riyadh	96	10.9
	Almadina Almonawra	25	2.8
	Eastern Region	20	2.3
	Albaha	18	2.1
	Aljouf	13	1.5
	Qassim	9	1.0
	Tabuk	9	1.0
	Jazan	7	0.8
	Hail	6	0.7
	Najran	10	1.1
	Northern Border	5	0.6
Occupation	Governmental employee	371	42.3
	Non-government employee	19	2.2
	Self-employed	40	4.6
	Students	220	25.1
	Housewife	170	19.4
	Retired	58	6.6
Economic status (Monthly Family Income in SAR)	Low (<2,000)	99	11.3
	Middle (2,000–4,999)	434	49.4
	High (≥5,000)	345	39.3

Table 2 reveals health profile, COVID-19 case contact, and medical field association among the study subjects. It displays that the majority (83.0%) of the study participants reported that they did not have any chronic diseases, and more than two-thirds (69.5%) of the respondents reported that they did not have any contact with COVID-19 cases. Around two-thirds (65%) of the study subjects reported that they did not have any association with the medical field.

RETRACTED

**Table 2:** Health profile, COVID-19 cases contact, and medical field association among the studied participants (*N* = 878).

**Variables**	**No. of subjects**	**Percentage (%)**
**Presence of chronic diseases**		
• NO	729	83.0
• YES	149	17.0
**Contact with COVID-19 Cases**		
• NO	610	69.5
• YES	268	30.5
[a] Family members	106	12.1
[b] Friends	79	9.0
[c] Neighbors	36	4.1
[d] Colleagues	28	3.2
[e] COVID-19 Cases	18	2.1
**Association with the medical field**		
• Not associated with the medical field	571	65.0
• Employees in the medical field	175	20.0
• Medical students	132	15.0

Table 3 shows the HRQOL status of the study participants during COVID-19 pandemic lockdowns. It represents that the highest mean of HRQOL domains was general health (55.31 ± 21.31), while the lowest mean of HRQOL domains was role limitation due to emotional problems (28.02 ± 22.98). The mean of MCS of the participants was 32.34 ± 25.30, which was lower than the mean of the PCS (41.65 ± 11.82).

**Table 3:** Health-related quality of life status of the participants during COVID-19 lockdown (*N* = 878).

**Health-related quality of life domains**	**Mean ± SD**	**Median**	**Minimum**	**Maximum**
General Health (GH)	55.31 ± 21.31	60	0	80
Physical Functioning (PF)	47.67 ± 23.77	66.67	0	66.67
Role-Physical (RP)	33.91 ± 21.48	50	0	50
Role-Emotional (RE)	28.02 ± 22.98	25	0	50
Bodily Pain (BP)	50.57 ± 20.36	60	0	80
Vitality (VT)	42.62 ± 21.02	33.33	0	83.33
Mental Health (MH)	46.83 ± 22.91	50	0	83.33
Social Functioning (SF)	35.58 ± 26.82	40	0	80
Physical Component Summary (PCS)/Physical HRQOL	41.65 ± 11.82	43.60	0.24	67.74
Mental Component Summary (MCS)/Mental HRQOL	32.34 ± 25.30	32.16	−24.64	91.77

Table 4 shows the perceived stress levels among the studied participants during COVID-19 lockdowns. It denotes that more than two-thirds (67.6%) of the study respondents reported that they had a moderate level of Stress during COVID-19 with mean ± SD (19.26 ± 3.27). The low level of Stress during COVID-19 was reported by 16.6% of the study subjects with mean ± SD (10.21 ± 2.50) whereas, the high level of Stress during COVID-19 was reported by 15.8% of them with mean ± SD (29.86 ± 2.88). It also shows that the overall mean of Stress during COVID-19 of the studied participants was (19.44 ± 6.39), and the variation coefficient among Stress during COVID-19 levels was also 28.6%.

RETRACTED

**Table 4:** Perceived stress levels among the participants during COVID-19 lockdown (*N* = 878).

**Perceived stress during COVID-19 level**	**No**.	**%**	**(Mean ± SD)**	**Total mean of stress during COVID-19**	**Variation coefficient**
Low level of stress	146	16.6	10.21 ± 2.50	19.44 ± 6.39	28.6%
Moderate level of stress	593	67.6	19.26 ± 3.27		
High level of stress	139	15.8	29.86 ± 2.88		

Table 5 displays the correlation between perceived COVID−19 total stress scores and HRQOL among the participants during the pandemic lockdown. It reveals the statistically significant negative relationship among total stress scores and HRQOL domains (GH, PF, RP, RE, BP, VT, SF, MH), as well as in physical component summary (PCS), and mental component summary (MCS).

**Table 5:** Correlation between perceived COVID−19 total stress scores and HRQOL among the participants during the pandemic lockdowns (*N* = 878).

**Health-related quality of life domains**	**Total stress scores *r*- value**	***p*-value**
General Health (GH)	−0.552**	0.000
Physical Functioning (PF)	−0.357**	0.000
Role-Physical (RP)	−0.471**	0.000
Role-Emotional (RE)	−0.528**	0.000
Bodily Pain (BP)	−0.540**	0.000
Vitality (VT)	−0.563**	0.000
Social Functioning (SF)	−0.414**	0.000
Mental Health (MH)	−0.628**	0.000
Physical Component Summary (PCS)	−0.212**	0.000
Mental Component Summary (MCS)	−0.673**	0.000

r, Pearson's correlation coefficient.

** *P significant at 0.01 level*.

Table 6 depicts the mean and difference among COVID-19 total stress, PCS, MCS, and socio-demographic characteristics of the study participants. It denotes that mean of total Stress during COVID-19 among older subjects who aged ≥60 years scored (20.39 ± 10.06) higher than other categories of age (19.59 ± 6.13), (19.06 ± 6.56), respectively, but the difference was not statistically significant. Males scored a significantly higher total mean of Stress during COVID-19 than females (F =12.413). Mean of COVID-19 overall stress among Saudi citizens were significantly lower than non-Saudi residents (*t* =2.778). Furthermore, single participants scored a significantly higher mean of Stress during COVID-19 than married (*t* =2.143). Retired citizens scored a significantly higher total mean of total stress than other participants during lockdown (*F* =6.176). Moreover, the participants whose monthly family income was insufficient scored a significantly higher total mean of Stress during COVID-19, and a lower total mean of MCS than other categories of economic status (F = 7.907), and (F =9.493), respectively. As age increased, there was decreased in total mean of the measures of physical HRQOL/PCS with statistically significant difference (t = 2.504). Married participants scored a significantly higher total mean of PCS, and MCS during lockdown than single (t = 3.731), (t =3.717), respectively. Females and Saudi participants scored a significantly higher total mean of the measures of mental HRQOL/MCS than males, and non-Saudi (t =2.758), and (t =3.349), respectively. Subjects who worked either in governmental or non-governmental sector scored a significantly higher total mean of PCS, and MCS than other categories of employment during lockdown (F =5.730), (F = 9.493), respectively.

RETRACTED

**Table 6:** Mean, and difference among COVID-19 total stress, PCS, MCS & sociodemographic characteristics of the study participants (*N* = 878).

**Socio-demographic Variables**	**Categories**	**Total stress**		**PCS**		**MCS**	
		**Mean**	**SD**	**Mean**	**SD**	**Mean**	**SD**
Age	18 to <40	19.59	6.13	42.94	11.96	31.77	25.00
	40 to <60	19.06	6.56	39.76	10.83	33.85	25.35
	≥60	20.39	10.06	33.81	14.35	27.39	31.64
F		**0.910**		12.413**		**1.098**	
Sex	Male	20.35	7.25	40.45	13.59	28.37	28.00
	Female	19.12	6.05	42.07	11.12	33.72	24.16
F		2.504**		**1.773**		2.758**	
Nationality	Saudi	19.18	6.46	41.80	11.86	33.53	25.50
	Non-Saudi	20.86	5.83	40.77	11.59	25.55	23.08
T		2.778**		**0.927**		3.349**	
Educational level	Primary & middle	18.29	5.64	40.72	11.68	33.07	21.43
	Secondary	19.39	6.90	39.43	12.27	34.34	24.97
	Graduation/PG	19.48	6.34	42.07	11.71	31.96	25.49
F		**0.403**		**2.777**		**0.488**	
Marital status	Married	19.08	6.49	43.55	12.44	34.78	24.77
	Unmarried	20.03	6.21	40.50	11.28	28.28	25.69
T		2.143*		3.731**		3.717**	
Occupation	Working personnel	18.59	6.41	43.38	12.46	35.77	24.35
	Housewife	19.54	6.28	41.89	10.96	33.25	24.48
	Student	20.60	7.47	40.48	12.56	30.86	28.12
	Retired	20.70	5.92	36.66	11.76	28.29	26.43
F		6.176**		5.730**		3.195*	
Family income	High (≥5,000)	18.50	6.22	42.74	11.31	35.79	24.27
	Middle (2,000–4,999)	19.80	6.37	41.13	12.14	31.59	25.35
	Low (<2,000)	21.10	6.73	40.12	11.89	23.59	26.48
F		7.907**		**2.743**		9.493**	

F, One-way analysis of variance (ANOVA) test-t = Independent sample t-test.

* p is significant at 0.05 level.

** *p is significant at 0.01 level*.

RETRACTED

Table 7 reveals mean and difference COVID-19 total stress, PCS, MCS, contact with the medical field, and COVID-19 cases among the study participants. The results indicate that subjects who reported that they had been diagnosed with a chronic disease scored a significantly higher total mean of Stress during COVID-19, and a lower total mean of PCS, and MCS than healthy participants (t =2.610), (t =4.688), and (t =2.712), respectively. COVID-19 patients scored a significantly higher total mean of Stress during COVID-19, and a lower total mean of PCS, and MCS than subjects who either have or have no contact history with COVID-19 cases. (F =17.943), (F =3.506), and (F =32.543), respectively. Subjects who reported that they worked in the medical field scored a significantly higher total mean of Stress during COVID-19 and PCS, and a lower total mean of MCS than subjects who did not work in the medical field. (t =3.150), (t =3.445), and (t =3.501), respectively.

**Table 7:** Mean and difference among COVID-19 total stress, PCS, MCS, relation with the medical field, and COVID-19 cases among the study participants (*N* = 878).

**Variable**	**Categories**	**Total Stress**		**PCS**		**MCS**	
		**Mean**	**SD**	**Mean**	**SD**	**Mean**	**SD**
Presence of chronic disease	Yes	20.68	7.30	37.56	12.82	27.23	25.93
	No	19.18	6.17	42.48	11.43	33.38	25.06
T		2.610**		4.688**		2.712**	
Contact with COVID-19 Cases	Yes	21.16	6.91	41.33	12.72	23.53	23.62
	No	18.62	5.85	41.99	11.29	36.59	24.67
	COVID-19 Patients	23.28	10.23	34.66	14.46	10.65	27.80
F		17.943**		3.506*		32.543**	
Medical field relation	Yes	20.36	5.67	43.51	12.31	28.29	24.97
	No	18.94	6.71	40.65	11.43	34.52	25.23
T		3.150**		3.445**		3.501**	

F, One-way analysis of variance (ANOVA) test t = Independent sample t- test.

* p, significant at 0.05 level.

** *p, significant at 0.01 level*.

## Discussion

The association of the current pandemic and its resultant restriction of activities is evident in the low mean scores of PCS and MCS in our sample (Tables 6, 7). In our study, the Mean PCS of 41.65 and Mean MCS of 32.34 is much lower (Table 3), as compared to the norms documented in a study conducted on US adults viz., Mean PCS of 50.12 and 50.04 as Mean MCS (19). Although there is no single study done in Saudi Arabia documenting HRQOL in the general population during the current COVID – 19 pandemic era. A study conducted among healthy female university students in Dammam using SF 12 reported mean PCS score of 69 and mean MCS score of 62, which are representative of the fair quality of life during non-pandemic times (20). The Quality of Life Scores in our study seems to be closer to those reported in patients of chronic diseases (Table 3), like Diabetes Mellitus and life-threatening events like Myocardial Infarction (21, 22). Moreover, the mental component scores are lower than physical component scores illustrating the disproportionately higher psychological association in the general population. This fact is reiterated on domain wise analysis which shows better scores in general health but the maximum limitation of the role due to emotional reasons (Table 3).

RETRACTED

This psychological component of pandemic association is further highlighted by perceived stress scores in our study with the majority (67.5%) of people reporting at least moderate levels of perceived stress and a substantial 15.8% reporting high perceived stress (Table 4). A similar study conducted in Colombia reported a 15% prevalence of high perceived stress during the current pandemic (23). Mean stress score in our study was 19.44 (Table 4), which is higher than that found by Limcaoco et al. (17.4) in their survey done in 41 countries (24), and by Chen et al. in Wuhan and surrounding areas where mean PSS scores in the general population and healthcare workers were found to be 14.8 and 16.8, respectively (25). Earlier researchers have consistently reported high-stress levels during current and past epidemics (24–27). The reasons for this stress may be multifactorial, like uncertainty about future and the disease, confusion and lack of information regarding the illness, loss of freedom, separation from family members, social isolation and taboo and many a times loss of wages due to lockdown as suggested by Brooks et al. (3).

The observed high-stress levels are evident in our study by a consistent inverse relationship between stress levels and all the domains of physical and mental functioning among the respondents (Table 5). A negative association between stress and HRQOL has been asserted by earlier researchers (28, 29).

In exploring important socio-demographic factors affecting stress and HRQOL during COVID - 19 pandemic, we found that men in our study reported significantly more stress levels and poorer MCS scores (Table 6). Classically, women have reported higher stress levels (30), as also reported during current epidemic in China by Qiu et al. (8), in Spain by Rodríguez-Rey et al. (31), in Austria by Pieh et al. (32) and in their systematic review by Luo et al. (33) Other researchers in Colombia could not report any significant impact between gender and psychological impact of COVID-19 (23). Relatively higher psychological influence in males than females in our study may be due financial crisis and problems related to their employment in the current situation. Other related factors were found to be unmarried status, lack of regular income, having a preexisting chronic disease and testing positive for COVID - 19, all corroborated by earlier researchers (33–35). Age and educational qualification were not found to be significantly associated with stress in our study (Table 6).

RETRACTED

Health care workers constitute a special at-risk group for stress in general and especially during epidemics. The current study reported higher mean stress scores among them during COVID-19 pandemic, when compared to stress scores in consultant physicians working in Kingdom of Saudi Arabia (17.0) during non-epidemic times (36). Similar high-stress levels in HCWs were reported in Korea (19.9) during MERS Cov epidemic (37), and in Hong Kong (18.0) during SARS outbreak (26). When compared to the general public, our study reveals significantly higher stress levels in healthcare workers (Table 7), which is congruent to the findings by Chen et al. (25). However; many researchers have failed to demonstrate a significant difference in the psychological impact of the epidemic on HCWs and the general population (24, 33). The root of the stress, as reported by Kang et al. may be “increased infection risk and improper protection from contamination, frustration, overburdened, favoritism, seclusion, patients with negative feelings, a lack of contact with family members, and sapping” (38).

## Strengths and Limitations of the Study

This study is the first study that investigates the association of COVID-19 with health-related quality of life in the general population of the KSA. Therefore, its results may help health authorities to plan preventive strategies that will aid in improving Health-Relate Quality of Life (HR-QOL) for future events. However, in interpreting the results of this study, some limitations should be considered. The study is limited by the use of an online questionnaire because of the inherent drawback of bias toward population having access to information technology. The study is also limited by the use of non-probability sampling technique. The method of sampling and data collection were chosen to materialize quick outreach to a maximum number of people during the period of restricted physical access in lockdown. Data collection was stopped when quarantine was lifted in KSA in order to fulfill the aim of the study. There is possibility of confounding in our study since all the analysis are unadjusted (not controlled for confounders such as pre-existing health conditions before COVID-19). As we do not have a PRE-COVID−19 measure of HRQoL or of general perceived stress, this cross-sectional nature of the survey is also a study limitation which further needs exploration in the form of randomized experiments in future. Another limitation is the smaller number of respondents aged 60 years & above in our study as compared to the age distribution of the general population of KSA. This can be attributed to the fact that the older individuals could not be approached because they do not frequently use various social media, twitter, e-mail etc. or don't use at all.

RETRACTED

## Conclusion

Majority subjects had a moderate level of stress related to COVID-19 during pandemic lockdowns. Stress during COVID-19 has a significant negative association on both physical and mental HRQOL in which MCS was significantly lower than PCS on the SF-12 scale. With the increase in the age of subjects, there was a significant decrease in physical HRQOL/PCS, and increase in total Stress during COVID-19, but this difference was insignificant. It is recommended that a longitudinal assessment is required to evaluate the effectiveness of stress management program, which can help the policymakers in formulating holistic interventions for affected individuals to alleviate the burden of the COVID-19 pandemic and its long-term sequelae.

## Data Availability Statement

The original contributions generated for the study are included in the article/supplementary material, further inquiries can be directed to the corresponding author/s.

## Ethics Statement

The study was approved by the Research Ethics Committee of King Khalid University. Informed consent to participate in the study was taken from all study subjects. Confidentiality of all personal information was ensured.

## Author Contributions

MH: instrumental in the concept, study design, preparing tool, analysis & drafting. AA: proposed the research design, overall supervision & final manuscript approval. WW: data acquisition, incorporated all the scientific intellect along with analysis. KM: prepared the final manuscript as per the required format of the journal. SM: drafted the primary manuscript & revised it critically. HA: responsible for preparing tool of the study, data entry, and statistical analysis. All authors contributed to the article and approved the submitted version.

## Conflict of Interest

The authors declare that the research was conducted in the absence of any commercial or financial relationships that could be construed as a potential conflict of interest.
